# Modelling the Role of Human Behaviour in Ebola Virus Disease (EVD) Transmission Dynamics

**DOI:** 10.1155/2022/4150043

**Published:** 2022-05-13

**Authors:** Sylvie Diane Djiomba Njankou, Farai Nyabadza

**Affiliations:** ^1^Department of Mathematics, University of Buea, PO Box 63, Buea, South West Region, Cameroon; ^2^Mathematics and Applied Mathematics Department, University of Johannesburg, Auckland Park, Kingsway Campus, Johannesburg, South Africa

## Abstract

The role of human behaviour in the dynamics of infectious diseases cannot be underestimated. A clear understanding of how human behaviour influences the spread of infectious diseases is critical in establishing and designing control measures. To study the role that human behaviour plays in Ebola disease dynamics, in this paper, we design an Ebola virus disease model with disease transmission dynamics based on a new exponential nonlinear incidence function. This new incidence function that captures the reduction in disease transmission due to human behaviour innovatively considers the efficacy and the speed of behaviour change. The model's steady states are determined and suitable Lyapunov functions are built. The proofs of the global stability of equilibrium points are presented. To demonstrate the utility of the model, we fit the model to Ebola virus disease data from Liberia and Sierra Leone. The results which are comparable to existing findings from the outbreak of 2014 − 2016 show a better fit when the efficacy and the speed of behaviour change are higher. A rapid and efficacious behaviour change as a control measure to rapidly control an Ebola virus disease epidemic is advocated. Consequently, this model has implications for the management and control of future Ebola virus disease outbreaks.

## 1. Introduction

Population growth and density in health risk areas of our societies do not facilitate the management of disasters whose number keeps growing as time evolves [1]. When a catastrophe arises, people can exhibit controlled behaviour which can take the form of intelligent and reasoned reactions [1]. However, panic or lack of knowledge can lead to a less controlled behaviour demonstrated by consideration or automated behaviour for example [1]. The efficacy of behaviour change can then be evaluated by the level of control in the behaviour of the affected population. During EVD outbreak of 2014 − 2016, the poor economic situation of the affected countries and some cultural beliefs impacted the level of control in the populations' behaviour, especially at the early stage of the epidemic.

High population mobility across porous borders, cultural beliefs, community resistance, strikes by health personnel, and messages fuelling despair are all behaviour-related factors listed by the World Health Organization (WHO) which contributed to the rapid and invisible spread of EVD [2]. Culturally meaningful behaviours such as washing and touching the deceased and bush-meat consumption practised in West Africa, unfortunately, helped to fuel EVD spread [3]. The disease was new to the unprepared health system of the affected countries which detected it three months after its onset in Guinea. So, a faster and more efficient behaviour change of the health authorities and the population would have greatly limited EVD spread and burden in West Africa [4, 5]. As a consequence, any EVD modelling framework that aims at controlling the disease must incorporate the efficacy and the speed of behaviour change and this is done in this manuscript. Mathematical models of Ebola virus disease (EVD) can be divided into two groups: models that do not account for infection due to EVD deceased and models that do. Models ignoring the deceased are classified as *SEIR* or *SIR* models; see for instance [6–12]. The incidence rate of these models is generally bilinear, i.e., of the form *βSI*. The formulation of such an incidence function increases the ease of analysing the models, including the global stability analysis of the fixed points using LaSalle's invariance principle [6, 10, 12]. However, neglecting the contribution of the deceased in the force of infection of EVD underestimates the number of Ebola cases [13].

Several models of EVD including a compartment for the deceased have been formulated and analysed; see for instance [14–19]. The mathematical analysis of the equilibria of such models mostly focuses on the determination of the reproduction number and local stability analysis of equilibria [17, 18]. The proof of the global stability of the equilibria is often neglected because of the nonlinearity of the incidence rate. Rivers et al. [15] modelled the impact of interventions on an epidemic of Ebola using a model that accounts for infection during funerals (*F*). The total population *N*, in this case, was made up of susceptibles (*S*), exposed (*E*), infected (*I*), hospitalized (*H*), and recovered (*R*) individuals. The incidence rate of the model which was given by (*βSI* + *β*_*H*_*SH* + *β*_*F*_*SF*)/*N*, accounted for infection during hospitalisation and burials. A similar structure of the incidence rate was used by Djiomba and Nyabadza [17] to investigate optimal control of EVD with educational campaigns, active case finding, and pharmaceutical interventions and Xia et al. [20] who modelled the transmission dynamics of Ebola in Liberia.

More complex incidence rates or forces of infection are found in disease models, especially those that incorporate behaviour change. Stopping a disease outbreak, in general, relies on the technical implementation of control strategies like vaccination, treatment, or educational campaigns. In the absence of treatment, a change in human behaviour will be the only hope to stop the disease spread. So, human behaviour remains the mainstay of any disease eradication, including EVD [21].

Psychology and anthropology are not the only domains interested in human behaviour. Mathematical modelling has also focused on the effects of human behaviour on various diseases' evolution; see for instance [21–25]. However, the quantification of human behaviour remains a challenge, and its effects on disease evolution are often represented by probabilities or by a modified incidence rate of the disease; see for instance [22]. Del Valle et al. [26] formulated a model to investigate the effects of behavioural changes in a smallpox attack. They assumed that individuals within a community change their behaviour and move from a normal active group to a less active group, reducing their average number of contacts, in response to a high prevalence of smallpox in the community. The per-capita transfer rate between compartments was modelled by the function *ϕ*_*i*_ = *a*_*i*_(*I*_*n*_ + *I*_*l*_)/(1 + *b*_*i*_(*I*_*n*_ + *I*_*l*_)) per day with *i* = *S*, *E*, *I* and where *n* = normally active, *l* = lessa ctive, and *a*_*i*_ and *b*_*i*_ being positive constants that modulate the rate of change. Behavioural change was thus taken to vary with the *ϕ*_*i*_ values and the transmission rate of smallpox. The force of infection for the normally active and less active was given by

(1) $$\begin{array}{c} \lambda_{j}=\frac{\gamma_{n}I_{n}+\gamma_{l}I_{l}+\gamma_{c}W}{\gamma_{n}A_{c}+\gamma_{l}A_{l}+\gamma_{c}A_{c}}, \end{array}$$

where *A*_*c*_ and *W* were, respectively, the confined and quarantined individuals, *j* = (*n*, *l*). They concluded that, besides the standard intervention procedure that would affect the extent and duration of a smallpox epidemic, the reduction in contacts of people in response to information about the epidemic was another contribution to smallpox control [26]. Wang X et al. [27] modelled the influence of human behaviour on cholera dynamics with a disease prevalence contact rate *β*_*i*_ = *a*_*i*_ − *b*_*i*_ *m*_*i*_(*I*), where *a*_*i*_ is the contact rate without considering the influence of human behaviour, *b*_*i*_ is the maximum reduced contact rate due to human behaviour, and *m*_*i*_(*I*) = *I*/*I* + *K*_*i*_, *i* = 1, 2, 3 where *K*_*i*_ is the half-saturation constant function. The contact rate was driven by a saturation function of the Michaelis Menten type. They concluded that human behaviour can reduce the endemic and epidemic levels, cholera spreading speeds, and the risk of infection [27]. Fractional derivatives are also recently used in disease modelling [28, 29]. A fractional model with behaviour is presented in [30]. This model uses fractional operators to investigate the asymptomatic behaviour of immunogenic tumour dynamics. The predictor-corrector method is adapted to the tumour-cell population dynamics and used to develop a tracking control method that helps to limit the growth of the tumour-cell population [30].

The impact of behaviour change on the spread of EVD with a linear force of infection has been done in [31]. Most of the EVD models that have been formulated to date are of the types *SEIR*, *SIR*, *SIRF*, *SEIRF*, and *SEIHRF*. In this paper, we consider a simple *SIRD* model, where *D* is the class of the deceased with a new nonlinear incidence function. In general, people abandon good behaviour when the perceived risk of a disease is reduced or because of limited funds to continue [32]. In the case of EVD, we assume that when the number of infected cases is well pronounced, the fear of contracting the disease obliges people to change their behaviour and a decline in the number of cases follows. Disease incidence or prevalence in a population has already been mentioned as a motivator of behaviour change during an epidemic for the case of influenza [26, 32]. Exponential functions have been suggested to represent the probability of disease transmission in the case of alertness to disease by Lio et al. [33]. Fast et al. [34] used a decreasing exposition probability, due to behaviour change between susceptible and infected individuals, to assess the role of social mobilisation in EVD control in Lofa.

The absence of treatment for EVD is a source of fear within the affected population and motivates a change in their behaviour leading to reduced disease transmission, especially when the number of infected cases reaches unexpected high values. In this model, we innovatively introduce a nonlinear force of infection that considers the efficacy and human behaviour change which were not considered in previous models [4, 5, 34]. EVD started in a rural area where it had been unnoticed for a few months, causing the force of infection to initially grow exponentially and later declined as the epidemic progressed [35]. Concave exponential functions are thus suitable to represent the force of infection. Among all the existing exponential functions, we propose a new Ricker-type function to represent the force of infection of our model. The function innovatively takes into consideration the efficacy and speed of behaviour change. It models the infection growth in the presence of behaviour change and the model fits better to EVD data from the two countries considered; see also [36]. The effective transmission rate of EVD is represented by the parameter *β* and the efficacy of behaviour change is represented by a parameter *p* (*p* ∈ [0, 1]) such that *p* = 0 corresponds to an uncontrolled behaviour that fuels EVD spread and *p* = 1 corresponds to a perfectly controlled behaviour that stops EVD spread. We also introduce a parameter *K* that represents the speed at which individuals change their behaviour. The parameter *K* helps to track how fast individuals change their behaviour in response to EVD. *K* = 0 corresponds to no behaviour change and greater values of *K* indicate a positive change in the affected population's behaviour. Total eradication of EVD corresponds to a zero force of infection for very high values of *K*(*K*⟶∞). We propose a force of infection given by

(2) $$\begin{array}{c} \lambda \left(t\right)=\beta \;\left(1-p\right)\left(I\left(t\right)+\varepsilon D\left(t\right)\right)\exp\left[-\left(I\left(t\right)+\varepsilon D\left(t\right)\right)K\right], \end{array}$$

where *ε* indicates the infectivity of the deceased when compared to that of the infected individuals, with *ε* > 1 and lim_*K*⟶∞_*λ* = 0.

This paper aims to study the dynamics of an EVD model with a nonlinear force of infection innovatively described by a Ricker function. We built the model with the assumption that behaviour change is motivated by disease incidence. We present the stability analysis of the model's steady states, and numerical simulations are used to confirm the modelling assumptions and to quantify the parameters modelling the efficacy and speed of behaviour change.

The paper is arranged as follows: in Section 2, we formulate the model.  Section 3 is reserved for the model analysis, and in Section 4, we focus on the steady states and their global properties.  Section 5 is reserved for the numerical simulations and the last section contains some concluding remarks.

## 2. Model Formulation and Equations

A deterministic model, consisting of individuals with different EVD statuses, is formulated to represent the population dynamics when there is a change of behaviour due to the high prevalence of the disease. Susceptible individuals (in compartment *S*) represent individuals that are at risk of contracting the infection through contact with the infected (in compartment *I*) and the deceased (in compartment *D*). Susceptible individuals are recruited into a heterogeneous population at a constant rate *Λ*. Infected individuals may recover at the rate *α* or may succumb to the Ebola virus and die at a rate *φ*. Individuals in each compartment are assumed to die naturally at a rate *μ*, and dead bodies of EVD-infected individuals deceased are disposed at a rate *ρ*. Dead bodies of infected individuals are assumed to be infectious. We thus assume here that infected individuals who do not die from EVD contribute to EVD spread and we set *δ* = *φ* + *μ* [37]. The total population size is given by

(3) $$\begin{array}{c} N\left(t\right)=S\left(t\right)+I\left(t\right)+R\left(t\right)+D\left(t\right). \end{array}$$

Figure 1 represents the movements between different classes, as their infection status with respect to the disease changes.

The governing equations that describe the dynamics of EVD as described are as follows:

(4) $$\begin{array}{c} \frac{\text{d}S\left(t\right)}{\text{d}t}=\Lambda -\left(\lambda \left(t\right)+\mu \right)\;S\left(t\right), \end{array}$$

(5) $$\begin{array}{c} \frac{\text{d}I\left(t\right)}{\text{d}t}=\lambda \left(t\right)\;S\left(t\right)-Q_{1}\;I\left(t\right), \end{array}$$

(6) $$\begin{array}{c} \frac{\text{d}R\left(t\right)}{\text{d}t}=\alpha \;I\left(t\right)-\mu \;R\left(t\right), \end{array}$$

(7) $$\begin{array}{c} \frac{\text{d}D\left(t\right)}{\text{d}t}=\delta \;I\left(t\right)-\rho \;D\left(t\right), \end{array}$$

where *Q*_1_ = (*α* + *δ*), with *S*(0) > 0, *I*(0) ≥ 0, *R*(0) ≥ 0, and *D*(0) ≥ 0.

## 3. Model Properties

### 3.1. Existence and Uniqueness of Solutions

The right-hand side of the system of differential equations (4)–(7) is made of Lipschitz continuous functions. According to Picard's existence theorem, with given initial conditions, the solutions of our system exist and they are unique [38].

**Theorem 1 .**

The system makes biological sense in the region

(8) $$\begin{array}{c} \Omega =\left\{\left(S\left(t\right),I\left(t\right),R\left(t\right),D\left(t\right)\right)\in {\mathbb{R}}_{+}^{4}:S\left(t\right)+I\left(t\right)+R\left(t\right)⩽\frac{\Lambda }{\mu }\text{ and }D\left(t\right)\leq \frac{\delta \;\Lambda }{\mu \;\rho }\right\}, \end{array}$$

which is attracting and positively invariant for the flow of system (4)–(7).

**Proof**

We set *H*(*t*) = *S*(*t*) + *I*(*t*) + *R*(*t*). By adding all the equations of system (4)–(6) we obtain

(9) $$\begin{array}{c} \frac{\text{d}H\left(t\right)}{\text{d}t}\leq \Lambda -\mu \;H\left(t\right). \end{array}$$

Using Gronwall inequality [39] and integrating (9), we obtain the following solution

(10) $$\begin{array}{c} H\left(t\right)\leq \left(H\left(0\right)-\frac{\Lambda }{\mu }\right)\exp\left[-\mu \;t\right]+\frac{\Lambda }{\mu },\forall t\geq 0. \end{array}$$

If *H*(0) ≤ *Λ*/*μ*, then the upper bound of *H*(*t*) is *Λ*/*μ* when *t*⟶∞. If *H*(0) ≥ *Λ*/*μ*, then *H*(*t*) decreases to *Λ*/*μ* when *t*⟶∞ and enters *Ω* or approaches *Ω* asymptotically.

Integrating (7) gives *D*(*t*) ≤ (*D*(0) − *Λ* *δ*/*ρ* *μ*)exp[−*ρ* *t*] + *Λ* *δ*/*ρ* *μ*, ∀*t* ≥ 0. If *D*(0) ≤ *Λ* *δ*/*ρ* *μ*, then *Λ* *δ*/*ρ* *μ* is the upper bound of *D*(*t*) when *t*⟶∞. If *D*(*t*) ≥ *Λ* *δ*/*ρ* *μ*, then *D*(*t*) decreases to *D*(*t*) ≥ *Λ* *δ*/*ρ* *μ* when *t*⟶∞ and enters *Ω*. Besides, any sum or difference of variables in *Ω* with positive initial values will remain in *Ω* or in a neighbourhood of *Ω*. Thus, *Ω* is bounded, positively invariant, and attracting for the flow of system (4)–(7).

### 3.2. Positivity of Solutions

**Theorem 2 .**

The existing solutions of our system (4)–(7) are all nonnegative.

**Proof**

We suppose that there exists $\hat{t}>0$ such that $S\left(\hat{t}\right)<0$. From the intermediate value theorem, there exists $t_{1}\in \left[0,\hat{t}\right]$ such that *S*(*t*_1_) = 0. From equation (4),

*S*(*t*) ≥ *S*(*t*_1_) exp[−(∫_0_^*t*^*λ*(*u*) *du* + *μ* *t*)] for all $t\in \left[t_{1},\hat{t}\right]$. *S*(*t*_1_) = 0 implies that *S*(*t*) ≥ 0 for *t* ≥ *t*_1_. Since $\hat{t}>t_{1}$, $S\left(\hat{t}\right)\geq 0$ and this contradicts the initial assumption. Thus, *S*(*t*) ≥ 0 for all *t* ≥ 0. The same principle is applied to *I*, *R*, and *D*, and from equation (5), we obtain *I*(*t*) ≥ *I*(*t*_1_) exp[−*Q*_1_ *t*], from equation (6), we obtain *R*(*t*) ≥ *R*(*t*_1_) exp[−*μ* *t*], and from equation (7), we obtain *D*(*t*) ≥ *D*(*t*_1_) exp[−*ρ* *t*]. We can then conclude that solutions of the system (4)–(7) are nonnegative.

## 4. Steady States and Global Properties

Equation (6) is redundant and the system of differential equations (4)–(7) can then be rewritten as

(11) $$\begin{array}{c} \frac{\text{d}S\left(t\right)}{\text{d}t}=\Lambda -\left(\lambda \left(t\right)+\mu \right)\;S\left(t\right), \end{array}$$

(12) $$\begin{array}{c} \frac{\text{d}I\left(t\right)}{\text{d}t}=\lambda \left(t\right)\;S\left(t\right)-Q_{1}\;I\left(t\right), \end{array}$$

(13) $$\begin{array}{c} \frac{\text{d}D\left(t\right)}{\text{d}t}=\delta \;I\left(t\right)-\rho \;D\left(t\right). \end{array}$$

Θ = {(*S*(*t*), *I*(*t*), *D*(*t*)) ∈ ℝ_+_^3^ : *S*(*t*) + *I*(*t*) ⩽ *Λ*/*μ* and *D*(*t*) ≤ *δ* *Λ*/*μ* *ρ*} is positively invariant and attracting since Θ ⊂ *Ω*.

Equations (11)–(13) admit a disease free equilibrium (DFE) denoted by *E*^0^ = (*Λ*/*μ*, 0, 0) and the next generation matrix method (see [40]) yields a reproduction number *R*_0_ given by *R*_0_ = *β* (1 − *p*)*Λ*/*μ*(1/*Q*_1_ + *ε* (*δ*/*ρ* *Q*_1_)). From the expression of the reproduction number, we can state that a more effective behaviour change reduces the number of secondary EVD infections.

The endemic equilibrium *E*^∗^ = (*S*^∗^, *I*^∗^, *D*^∗^) is given by

(14) $$\begin{array}{c} S^{*}=\frac{\Lambda \;\rho }{\left(\mu \;\rho +\beta \;\left(1-p\right)I^{*}\;\left(\delta \;\varepsilon +\rho \right)\exp\left[-I^{*}\left(1+\varepsilon \delta /\rho \right)K\right]\right)}, \end{array}$$

(15) $$\begin{array}{c} D^{*}=\frac{\delta }{\rho }\;I^{*}. \end{array}$$

*I* ^∗^ is solution of the equation

(16) $$\begin{array}{c} \beta \;\left(1-p\right)S^{*}\;I^{*}\;\left(1+\frac{\delta \;\varepsilon }{\rho }\right)\exp\left[-I^{*}\;\left(1+\frac{\delta \;\varepsilon }{\rho }\right)\;K\right]-Q_{1}\;I^{*}=0, \end{array}$$

obtained by substituting equations (14) and (15) into equation (12).

We set *M*(*I*^∗^) = *β* (1 − *p*) *S*^∗^ *I*^∗^ (1 + *δ* *ε*/*ρ*)exp[−*I*^∗^ (1 + *δ* *ε*/*ρ*)*K*] − *Q*_1_ *I*^∗^ and find the roots in Θ of the function *M*. However, the exponential function does not facilitate the algebraic resolution of equation (16). We first rewrite the function *M* as *M*(*I*^∗^) = (Γ(*I*^∗^) − *Q*_1_) *I*^∗^ where Γ(*I*^∗^) = *β* (1 − *p*) *S*^∗^ (1 + *ε* (*δ*/*ρ*))exp[−*I*^∗^ (1 + *δ* *ε*/*ρ*)*K*] and *I*^∗^ = 0 is a root of *M* which corresponds to the DFE. The endemic equilibrium point (*I*^∗^) is the solution of Γ(*I*^∗^) = *Q*_1_. We have

(17) $$\begin{array}{c} \frac{d\Gamma \left(I^{*}\right)}{dI^{*}}=-\frac{\beta \;\left(1-p\right)\;\Lambda \;{\left(\delta \;\varepsilon +\rho \right)}^{2}\;\left(\beta \;\left(1-p\right)+\mu \;K\exp\left[I^{*}\left(1+\delta \;\varepsilon /\rho \right)K\right]\right)}{{\left(I^{*}\;\beta \left(1-p\right)\;\left(\delta \;\varepsilon +\rho \right)+\mu \;\rho \exp\left[I^{*}\left(1+\delta \;\varepsilon /\rho \right)K\right]\right)}^{2}}<0, \end{array}$$

and Γ(0) = *R*_0_ *Q*_1_ and lim_*I*^∗^⟶∞_Γ(*I*^∗^) = 0.

So Γ(*I*^∗^) is a monotone decreasing and positive function which intercepts the line *y* = *Q*_1_ only once when *R*_0_ > 1. In fact, the graph of Γ can intercept the line *y* = *Q*_1_ if Γ(0) ≥ *y*(0) because Γ is a decreasing function. Since Γ(0) = *R*_0_ *Q*_1_, Γ(0) is above *Q*_1_ when *R*_0_ > 1. If *R*_0_ < 1, Γ(0) is below *Q*_1_, implying that we have no endemic equilibrium. We can then conclude that our model has a unique endemic equilibrium point when *R*_0_ > 1.

We use the parameter values obtained by the fitting process in Figure 2(a) to illustrate the existence of a unique endemic equilibrium point in Figure 3.

Note that any *I*, *D* ∈ Θ, inequality (21) is valid i.e.

(18) $$\begin{array}{c} \exp\left[-\psi \right]\leq \exp\left[-\left(I+\varepsilon D\right)K\right]\leq 1,\text{where }\psi =\frac{\Lambda }{\mu }\left(1+\in \frac{\delta }{\rho }\right)K. \end{array}$$

### 4.1. The disease free equilibrium

**Theorem 3 .**

The unique EE exists when *R*_0_ > 1, and when inequality (18) holds, it is globally asymptotically stable.

**Proof**

To prove the global stability of the EE, we set *F* as a candidate Lyapunov function and we give conditions under which $\dot{F}$ is nonpositive.

(19) $$\begin{array}{c} F=\left(S-S^{*}-S^{*}\ln\left(\frac{S}{S^{*}}\right)\right)+A\;\left(I-I^{*}-I^{*}\ln\left(\frac{I}{I^{*}}\right)\right)+G\;\left(D-D^{*}-D^{*}\ln\left(\frac{D}{D^{*}}\right)\right), \end{array}$$

where *A* and *G* are positive constants to be calculated with *F*(*E*^∗^) = 0.

The right-hand side of system (11)–(13) at equilibrium yields

(20) $$\begin{array}{c} \Lambda =\left(\beta \;\left(1-p\right)\left(I^{*}+\varepsilon D^{*}\right)\exp\left[-\left(I^{*}+\varepsilon D^{*}\right)K\right]+\mu \right)S^{*}, \end{array}$$

(21) $$\begin{array}{c} Q_{1}=\frac{S^{*}}{I^{*}}\;\beta \;\left(1-p\right)\left(I^{*}+\varepsilon D^{*}\right)\exp\left[-\left(I^{*}+\varepsilon D^{*}\right)K\right], \end{array}$$

(22) $$\begin{array}{c} D^{*}=g\;I^{*}, \end{array}$$

where *g* = *δ*/*ρ*.

The derivatives of *F* with respect to each state variable are

(23) $$\begin{array}{c} \frac{\partial \;F}{\partial S}=\left(1-\frac{S^{*}}{S}\right),\\ \frac{\partial \;F}{\partial I}=A\;\left(1-\frac{I^{*}}{I}\right),\\ \frac{\partial \;F}{\partial D}=G\;\left(1-\frac{D^{*}}{D}\right),\\ \frac{\partial^{2}\;F}{\partial S^{2}}=\left(\frac{S^{*}}{S^{2}}\right),\\ \frac{\partial^{2}\;F}{\partial I^{2}}=A\;\left(\frac{I^{*}}{I^{2}}\right),\\ \frac{\partial^{2}\;F}{\partial D^{2}}=G\;\left(\frac{D^{*}}{D^{2}}\right). \end{array}$$

*E* ^∗^ is then the unique critical point of *F*, and since the second derivative of *F* is positive at any point of Θ, the Lyapunov function *F* is concave up and the unique endemic equilibrium point is the global minimum of *F*.

The derivative of *F* with respect to time *t*, denoted by $\dot{F}$, is

(24) $$\begin{array}{c} \dot{F}=\left(1-\frac{S^{*}}{S}\right)\;\dot{S}+A\;\left(1-\frac{I^{*}}{I}\right)\;\dot{I}+G\;\left(1-\frac{D^{*}}{D}\right)\;\dot{D}. \end{array}$$

Considering the system of equations (11)–(13) together with inequality (??) and the fact that *E*^∗^ is the global minimum of *F*, we obtain

(25) $$\begin{array}{c} \dot{F}\leq \left(1-\frac{S^{*}}{S}\right)\left(\Lambda -\left(\beta \;\left(1-p\right)\left(I+\varepsilon \;D\right)\exp\left[-\psi \right]+\mu \right)S\right)+A\;\left(1-\frac{I^{*}}{I}\right)\left(\beta \;\left(1-p\right)\left(I+\varepsilon \;D\right)S-Q_{1}\;I\right)+G\left(1-\frac{D^{*}}{D}\right)\left(\delta \;I-\rho \;D\right). \end{array}$$

We set

(26) $$\begin{array}{c} x=\frac{S}{S^{*}},\\ y=\frac{I}{I^{*}},\\ u=\frac{D}{D^{*}}, \end{array}$$

and rewrite (25) as

(27) $$\begin{array}{c} \dot{F}\leq -\mu \;\frac{{\left(S-S^{*}\right)}^{2}}{S}+\beta \;\left(1-p\right)\;I^{*}L\left(x,y,u\right), \end{array}$$

where

(28) $$\begin{array}{c} L\left(x,y,u\right)=\left(1-\frac{1}{x}\right)S^{*}\left(\left(1-x\;y\;\exp\left[-\psi \right]\right)+g\;\varepsilon \;\left(1-u\;x\;\exp\left[-\psi \right]\right)\right)+A\;\left(1-\frac{1}{y}\right)S^{*}\;\left(y\;\left(x-1\right)+\varepsilon \;g\;\left(u\;x-y\right)\right)+\frac{G\;\delta }{\beta \;\left(1-p\right)}\left(1-\frac{1}{u}\right)\left(y-u\right). \end{array}$$

The expression of *L* is obtained by replacing *Λ*, *Q*_1_, and *g* in equation (25) by their expressions from equations (21).

Expanding the expression of *L*(*x*, *y*, *u*) from system (28) and grouping the coefficients with the same variable give

(29) $$\begin{array}{c} L\left(x,y,u\right)=\frac{G\;\delta }{\beta \;\left(1-p\right)}+S^{*}\;\left(A+1\right)+S^{*}\;\varepsilon \;g\;\left(A+1\right)+y\;\left(\frac{G\;\delta }{\beta \;\left(1-p\right)}+S^{*}\;\left(\exp\left[-\psi \right]-A\right)-\varepsilon \;g\;A\;S^{*}\right)+u\;\left(-\frac{G\;\delta }{\eta \;\left(1-p\right)}+\varepsilon \;g\;S^{*}\exp\left[-\psi \right]\right)+\frac{y}{u}\left(-\frac{G\;\delta }{\beta \;\left(1-p\right)}\right)+\frac{1}{x}\left(-S^{*}-\varepsilon \;g\;\exp\left[-\psi \right]S^{*}\right)-x\;A\;S^{*}+x\;y\left(-S^{*}\;\exp\left[-\psi \right]+A\;S^{*}\right)+u\;x\;\left(-\varepsilon \;A\;g\;S^{*}+\varepsilon \;A\;g\;\exp\left[-\psi \right]S^{*}\right)+\frac{u\;x}{y}\left(-A\;g\;S^{*}\;\varepsilon \right). \end{array}$$

Since we already have −*μ* ((*S* − *S*^∗^)^2^/*S*) ≤ 0 from the expression of $\dot{F}$, it remains to prove that *L* ≤ 0 in order to get $\dot{F}\leq 0$.

From the expression of *L* in (29), we will first set the terms containing variables and with nonnegative coefficients to zero in order to get rid of the positive and nonconstant part of *L*. The coefficients of *y*, *u*, *x* *y*, and *u* *x* are thus set to zero and solved for *A* and *G*. We obtain

(30) $$\begin{array}{c} A=\exp\left[-\psi \right],G=\frac{\varepsilon \;g\beta \;\left(1-p\right)}{\delta }S^{*}\exp\left[-\psi \right],\\ L\left(x,y,u\right)=\frac{G\;\delta }{\beta \;\left(1-p\right)}\;\left(1-\frac{y}{u}\right)+\varepsilon \;g\;S^{*}\;\left(A\;\left(1-\frac{1}{x}\right)+1-\frac{u\;x}{y}\right)+\left(A\left(1-x\right)+1-\frac{1}{x}\right)S^{*}. \end{array}$$

So *L* is negative and will be equal to zero if *x* = *y* = *u* = 1 which is in the set

(31) $$\begin{array}{c} C=\left\{\left(S,I,D\right)\text{: }S=S^{*},I=I^{*},D=D^{*}\right\}. \end{array}$$

LaSalle's extension implies that each solution which intersects ℝ_+_^3^ limits to the endemic equilibrium and *E*^∗^ is globally asymptotically stable on Θ (see [41]).

Global stability of the EE indicates that EVD persists as long as the value of the reproduction number is greater than one. Programs aiming at eradicating EVD should limit the disease transmission in such a way that the value of the reproduction number remains less than one.

## 5. Numerical Simulations

### 5.1. Model Validation

We fit the number of new EVD cases *I*(*t*) from our model to data from Liberia and Sierra Leone [42].  Table 1 gives the number of new Ebola cases recorded in two countries. The values of the parameters estimated through the least-squares fitting process are given in Table 2. A comprehensive description of the least-squares fitting method is given in [19].

Figures 2(a) and 4(a) show that our model closely fits to the data and indicate that behaviour change during the EVD outbreak of 2014 − 2016 was motivated by an increased number of EVD cases. They also show that an efficacious behaviour change was necessary to stop EVD spread. Figures 2(b) and 4(b) show a poor fit of the model to data from Liberia and Sierra Leone when there is a slow and inefficacious behaviour change, resulting in an uncontrolled behaviour during EVD epidemic (*K* = 0.005, *p* = 0). The controlled or efficacious behaviour adopted by populations in order to limit EVD spread consisted of practising careful hygiene, avoiding contact with infected animals and humans, collaborating with case tracking, not fleeing from isolation areas, safely burying those who died from EVD, etc. [17, 43]. Figures 2(b) and 4(b) predict an increased number of infected individuals (represented by the continuous line) when compared to Figures 2(a) and 4(a), thus overestimating the number of EVD cases. This increase is due to a slower and nonefficacious behaviour change that caused the EVD epidemic to last longer and to claim more human lives. Behaviour change should be advocated at the beginning of an epidemic, to limit the death toll of the disease and its spread.

The values of the estimated parameters in Table 2 yield a reproduction number equal to 1.71 in Liberia and 2 in Sierra Leone when there is a rapid and controlled change in human behaviours. These values are comparable to those obtained by several authors. Rivers et al. [15] found that the value of the reproduction number for the two countries on an average is 2.2. Althaus [44] found *R*_0_ = 1.59 for Liberia and *R*_0_ = 2.53 for Sierra Leone in 2014. Xia et al. [20] found *R*_0_ = 2.02 for Liberia when investigating the different transmission routes of EVD. Chowell and Nishiura [11] estimated the value of the reproduction number between 1 and 2 in Liberia and Sierra Leone, from March to August 2014. The difference between the estimated and cited values of the reproduction number might come from the fact that they are calculated during different periods of EVD epidemics and the models built by the authors have different structures and integrate different control measures in some instances.

Behaviour change influenced several factors such as the EVD transmission rate, death rate, recovery rate, and even the burial rate of the deceased. Avoiding contact between susceptible and infected individuals, for example, contributed to a reduction in the transmission rate of EVD. This explains why the value of *β* estimated in Table 2 when controlled behaviour is considered is less than the one from the fitting with slow behaviour change and uncontrolled behaviour. Some researchers concluded that the transmission rate of EVD is higher without behaviour change [15, 20]. The recovery rate and death rate of EVD are influenced by the collaboration between populations and authorities through active case finding or hospitalisation for example. Recovering from EVD without treatment was very rare and can explain the low values of *α* estimated in Table 2. The case fatality rate of the last EVD epidemic was greater than 50% [15, 20, 37], indicating a high risk of death for EVD patients. This supports the estimated values of *δ* in Table 2 for both countries. In [45], the values of *δ* are greater without a controlled behaviour, highlighting the importance of adopting disease reducing behaviours like visiting the appropriate health centres to receive pharmaceutical interventions that help to increase the chances of recovering from EVD. Dead bodies of EVD deceased are twice more infectious than the living infected individuals according to the estimation of *ε*. Some authors found that this infectivity could be even four times higher for the deceased [20]. Quick and safe burials of EVD deceased have helped to limit EVD spread, and the high values of *ρ* from Table 1 indicate that a high burial rate helped to limit the disease spread. The estimated values of *p* indicate that a highly efficacious behaviour change, adapted to health authorities' instructions, for example, was necessary to halt EVD spread. The estimated values of *K* indicate how fast a behaviour change occurred during the last EVD epidemic in Liberia and Sierra Leone. However, these values are low and this implies that behaviour change was a slow process during the outbreak. This could explain the long duration of the outbreak and its extent in terms of the number of deaths. Cultural beliefs and poor economic conditions build mistrust between rural populations and authorities in West Africa [3]. This situation led to a slow application of instructions from authorities during the outbreak. So, building confidence and improving people's living conditions is essential in motivating people to quickly react in case of an epidemic of EVD.

### 5.2. Sensitivity Analysis

The reproduction number *R*_0_ is made of different parameters and their correlations to *R*_0_ differ as well. Sensitivity analysis helps to assess the variability in the model predictions introduced by uncertainty in the parameters value [46]. We use Latin hypercube sampling (LHS) and partial correlation coefficient (PRCC) to explore the parameter space of the model with 1000 simulations [47]. We choose a uniform distribution to implement LHS sampling scheme. The PRCC value for a specific parameter is a Pearson correlation coefficient for the residuals from two regression models [46]. The most important parameters have a PRCC value greater than 0.5 or less than −0.5.  Figure 5 represents the sensitivity analysis of *R*_0_.

We observe in Figure 5 that the parameters with the most important positive correlations to *R*_0_ are *δ*, *Λ*, and *β* and those with the negative correlations are *ρ*, *μ*, and *p*. The results show that when the transmission rate and death rate of EVD increase, the number of new infections increases since the deceased and infected individuals are both infectious. When the recruitment rate is increased, more individuals are exposed to the Ebola virus and this increases their chances of contracting the virus and contributes to the disease's spread. Natural death reduces the size of the population and thus limits the number of people who might be infected by EVD. Disposing of the corpses of EVD deceased rapidly and safely stops contamination during funerals and reduces the potential number of EVD cases. The negative correlation between *R*_0_ and *p* is certainly because adopting a controlled behaviour that limits or stops EVD spread reduces the reproduction number and is represented by an increase of the value of *p*.

## 6. Conclusion

The global stability analysis of the steady states of a model of EVD with a nonlinear incidence function is presented in this paper. The global stability of equilibria is presented through suitably chosen Lyapunov functions. The nonlinear incidence function is chosen to represent the influence of human behaviour on EVD evolution. Data from Liberia and Sierra Leone are used in the fitting process whose results show that the model closely describes the evolution of EVD with human behaviour. Parameters obtained in the fitting process support the assumptions made in the development of the model that behaviour change is motivated by disease prevalence. As soon as an epidemic starts, individuals affected should trust the authorities and do as instructed to avoid deaths and disasters due to a slow reaction.

The work presented in this paper is not without shortcomings. The modelling of human behaviour through any mathematical function is a challenge as human behaviour is complex and unpredictable. A stochastic version of the incidence function may be worth looking at as an alternative albeit the challenges associated with its formulation and the mathematical analysis. The use of individual-based models or network models could potentially solve the inadequacies of dealing with deterministic models. We still however argue that this model presents some interesting mathematical results on the global stability of an EVD model with human behaviour and a nonlinear incidence rate.

The theory of fractional calculus is often used for modelling purposes in general [48–50]. In disease modelling, in particular, fractional derivatives which are used in modelling the dynamics of an infectious disease like COVID-19 [51] could also be applied to Ebola virus disease models in future works.

## Figures and Tables

**Figure 1:** Flow diagram of the model. This four-compartmental diagram describes the progression of individuals during an EVD outbreak and also indicates the rates at which people move from one compartment to another.

**Figure 2:** Curve fitting with data collected from Liberia. The fitting process considers a controlled behaviour in (a) and an uncontrolled behaviour in (b). Parameters such as the efficacy and speed of behaviour change are increased in (a) to investigate how they affect the quality of the fit.

**Figure 3:** Intersection of *Q*_1_ and Γ(*I*^∗^). The fitting process in Figure 2(a) yields parameter values used to numerically illustrate the existence of a unique endemic equilibrium point.

**Figure 4:** Curve fitting with data collected from Sierra Leone. The fitting process considers a controlled behaviour in (a) and an uncontrolled behaviour in (b). Parameters such as the efficacy and speed of behaviour change are increased in (a) to investigate how they affect the quality of the fit.

**Figure 5:** Tornado plot of the sensitivity analysis of *R*_0_. This figure represents the correlation coefficient of each parameter which constitutes the reproduction number *R*_0_. The aim is to compare these correlations and determine the most important.

**Table 1:** Data from Liberia and Sierra Leone as indicated by the Centers for Disease Control and Prevention website. Each month is labelled by the first three letters of his name on the Egyptian calendar. Nav stands for not available.

Year	2014										2015									
Month	Mar	Apr	May	Jun	Jul	Aug	Sept	Oct	Nov	Dec	Jan	Feb	Mar	Apr	May	Jun	Jul	Aug	Sept	Oct
Data of Liberia	2	3	5	76	166	1142	1317	477	200	145	30	12	2	0	0	0	0	0	0	0
Data of Sierra Leone	Nav	Nav	20	205	369	770	1233	1649	2499	1579	864	358	252	49	40	46	26	5	0	0

**Table 2:** Estimated values of the parameters for each country.

Parameters	Liberia		Sierra Leone	
	Controlled behaviour	Uncontrolled behaviour	Controlled behaviour	Uncontrolled behaviour
*Λ*	26	150	26	150
*δ*	0.55	0.7	0.5	0.6
*ρ*	0.9	0.98	0.99	0.76
*μ*	0.0205	0.2117	0.0285	0.1523
*ε*	2.25	2	2	2
*β*	0.0047	0.0091	0.0047	0.0088
*α*	0.012	0.012	0.012	0.012
*p*	0.82	0	0.818	0
*K*	0.003	0.005	0.003	0.005

## Data Availability

Data are available at https://apps.who.int/gho/data/node.ebola-sitrep.ebola-country-GIN-20141112?lang=en.
